# Regulation of CDKN2B expression by interaction of Arnt with Miz-1 - a basis for functional integration between the HIF and Myc gene regulatory pathways

**DOI:** 10.1186/1476-4598-13-54

**Published:** 2014-03-11

**Authors:** Reidun Aesoy, Katarina Gradin, Kathrine S Aasrud, Erling A Hoivik, Jorge L Ruas, Lorenz Poellinger, Marit Bakke

**Affiliations:** 1 Department of Biomedicine, University of Bergen, Jonas Lies vei 91, N-5009 Bergen, Norway; 2 Department of Cell and Molecular Biology, Karolinska Institutet, S-171 77 Stockholm, Sweden; 3 Cancer Science Institute Singapore, National University of Singapore, Singapore 117456, Republic of Singapore; 4 Present address: Department of Physiology and Pharmacology, Karolinska Institutet, S-171 77 Stockholm, Sweden

**Keywords:** Helix-loop-helix transcription factors, Hypoxia, Hypoxia-inducible factor (HIF), Myc, Arnt, CDKN2B, Miz-1

## Abstract

**Background:**

Hypoxia- and Myc-dependent transcriptional regulatory pathways are frequently deregulated in cancer cells. These pathways converge in many cellular responses, but the underlying molecular mechanisms are unclear.

**Methods:**

The ability of Miz-1 and Arnt to interact was identified in a yeast two-hybrid screen. The mode of interaction and the functional consequences of complex formation were analyzed by diverse molecular biology methods, in vitro. Statistical analyses were performed by *Student’s t-test* and *ANOVA*.

**Results:**

In the present study we demonstrate that the aryl hydrocarbon receptor nuclear translocator (Arnt), which is central in hypoxia-induced signaling, forms a complex with Miz-1, an important transcriptional regulator in Myc-mediated transcriptional repression. Overexpression of Arnt induced reporter gene activity driven by the proximal promoter of the cyclin-dependent kinase inhibitor 2B gene (*CDKN2B*), which is an established target for the Myc/Miz-1 complex. In contrast, mutated forms of Arnt, that were unable to interact with Miz-1, had reduced capability to activate transcription. Moreover, repression of Arnt reduced endogenous CDKN2B expression, and chromatin immunoprecipitation demonstrated that Arnt interacts with the *CDKN2B* promoter. The transcriptional activity of Arnt was counteracted by Myc, but not by a mutated variant of Myc that is unable to interact with Miz-1, suggesting mutually exclusive interaction of Arnt and Myc with Miz-1. Our results also establish *CDKN2B* as a hypoxia regulated gene, as endogenous CDKN2B mRNA and protein levels were reduced by hypoxic treatment of U2OS cells.

**Conclusions:**

Our data reveal a novel mode of regulation by protein-protein interaction that directly ties together, at the transcriptional level, the Myc- and hypoxia-dependent signaling pathways and expands our understanding of the roles of hypoxia and cell cycle alterations during tumorigenesis.

## Introduction

Hypoxia inducible factors (HIFs) are transcriptional regulators essential for cellular responses to low O_2_ levels (hypoxia). The HIFs belong to the family of helix-loop-helix (HLH)-*Per-Arnt-Sim* (PAS) factors, which act as sensors for environmental and developmental signals. HIF complexes consist of an O_2_-regulated Hifα-subunit and the ubiquitously expressed dimerization partner protein, the aryl hydrocarbon receptor nuclear translocator (Arnt). Arnt is essential in multiple cellular regulatory pathways, as it functions as an obligate heterodimerization partner for many HLH-PAS proteins. Three Hifα-subunits are known, of which Hif1α and Hif2α are the best characterized. (Hif1α and Hif2α will commonly be referred to as Hifα in this paper). In the canonical hypoxic transcriptional response, Hif1α and Hif2α are stabilized at low O_2_ tension and translocate to the nucleus where they bind to hypoxia response elements (HREs) together with Arnt (reviewed in [1,2]). HREs are present in many hypoxia-regulated genes, as in for instance genes that promote cell survival at low- O_2_ conditions (e.g. vascular endothelial growth factor and glucose transporter-1, which induce angiogenesis and glycolysis respectively [3]). However, Hif1α also confers transcriptional repression, and is then typically indirectly recruited to target genes via protein interactions [4,5].

Myc directs changes in metabolism, protein synthesis and cell proliferation through its transcriptional activity [6]. In the course of transcriptional activation, Myc interacts with its partner Max at E-box elements within target gene promoters. In contrast, when Myc acts as a transcriptional repressor, it interacts indirectly with DNA through other transcription factors [7]. One such factor is Miz-1 (Myc-interacting zinc finger protein 1). Miz-1 typically interacts with initiator (INR)-like elements in close proximity to the transcriptional start site and activates expression of target genes. Some of the first targets identified for Miz-1 were genes encoding cyclin-dependent kinase (CDK) inhibitors (CDKIs) (e.g. *CDKN1A* and *CDKN2B*), and consequently Miz-1 inhibits cell cycle progression [8-10]. When Myc-levels rise within the cell, Myc, in complex with Max, binds to Miz-1 and displaces the co-activator p300 with subsequent loss of the transcriptional potential of Miz-1 [10]. Although Miz-1 was first identified as a Myc-interacting protein and inducer of cell cycle arrest [11], Miz-1 also promotes cell survival and proliferation in some cellular contexts [12,13]. Myc is the only bHLH factor hitherto known to interact with Miz-1, but Miz-1 interacts with many other types of proteins, and functions of Miz-1 that are independent of Myc have been recognized [14-17].

Myc and hypoxia dependent transcriptional signaling is frequently deregulated in cancer cells, and importantly, these pathways are closely integrated in several processes that are altered in tumors (e.g. carbon metabolism, protein synthesis and cell cycle progression [18,19]). Myc and HIFs converge on many gene promoters, and can either act in concert or counteract each other. Generally, the literature suggest that Hifα enhances Myc action on genes that are involved in angiogenesis and glycolysis, but opposes Myc on promoters controlling the expression of genes implicated in DNA repair, mitochondrial biogenesis and cell proliferation [20]. For example, Hif1α displaces c-Myc from Sp-1 leading to repression of DNA repair genes [4,5]. With regard to genes controlling cell cycle progression, the scenario is more complex, and the underlying mechanisms less well understood. Collectively, the existing literature strongly indicates that the final transcriptional outcome will vary depending on the hypoxic environment and on cellular and promoter context [1,21]. Moreover, the transcriptional response and subsequent effects on cell cycle progression most likely also depend on whether the cell expresses predominantly Hif1α or Hif2α [22]. In this study we present a molecular interaction that might function as a molecular hub that unites hypoxia- and Myc-dependent signaling. We demonstrate that Arnt is an interaction partner for Miz-1, and that Arnt has a functional role in the regulation of *CDKN2B*, a known target for the Myc/Miz complex.

## Results

### Arnt and Miz-1 interact

We initially observed the interaction between Miz-1 and Arnt in a yeast two-hybrid screen where a deletion mutant of Arnt lacking the transactivation domain (ArntΔQ; amino acid (aa) 1–618) was found to interact with the C-terminal part of Miz-1 (aa 470–794; data not shown). Diverse Arnt constructs (schematically presented in Figure 1A) were tested for their ability to interact with Miz-1 in mammalian cells. Cos-1 cells were transiently transfected with Arnt/Flag and Miz-1/GFP and, as demonstrated in Figure 1B (upper panel), Arnt precipitated together with Miz-1 suggesting that these two factors interact in vivo. For the interaction to occur, the basic HLH (bHLH) domain of Arnt was required, but not the PAS domain (Figure 1B, upper panel). Complex formation between Miz-1 and Myc requires amino acids V393, V394, K397 and S405 in helix II of the HLH-domain of Myc [14]. Alignment of Myc and Arnt demonstrated that with regard to charge and hydrophobicity, a similar interactions surface is present in helix II of Arnt by the amino acids L114, T115, R118 and S126 (Figure 1A). Mutation of amino acid T115 and S126 (2xmut; T115D/S126A) decreased the ability of Arnt to interact with Miz-1, and mutation of all four amino acids (4xmut; L114A/T115D/R118G/S126A) reduced complex formation below the detection limit of the assay (Figure 1B, upper panel), pointing to a similar mode of interaction between Arnt and Miz-1 as between Myc and Miz-1. Control experiments demonstrated comparable expression levels of wt Arnt and the different mutants (Figure 1B, middle panel), and moreover that Miz-1 was precipitated at similar levels in all samples, although slightly less in lanes 1 and 6 (Figure 1B, lower panel). Experiments designed to map the domain(s) of Miz-1 involved in complex formation failed, presumably because the different deletion constructs exhibited different cellular localization (i.e. cytoplasmic, nuclear or perinuclear; data not shown). Work by Peukert and colleagues indicate that Miz-1 lacks a functional nuclear localization signal, however they found that overexpression of Myc induces a redistribution of Miz-1 from the cytoplasm to the nucleus [11]. To investigate whether Arnt would alter the localization of Miz-1, Arnt/CFP and Miz-1/Flag were expressed in HEK293 cells. Consistent with previous reports, Arnt/CFP localized exclusively to the nucleus whereas Miz-1/Flag was distributed diffusely throughout the cell when expressed singlehandedly (Figure 1C) [11,23,24]. Notably, in cells where Arnt/CFP and Miz-1/Flag were co-expressed, Miz-1/Flag was repositioned from the cytoplasm to the nucleus (Figure 1C). Although co-localization of the two proteins in HEK293 cells was not observed under these experimental conditions, this result suggests that overexpression of Arnt induces a cellular redistribution of Miz-1 and indicates a functional significance for the Miz-1/Arnt complex.

**Figure 1:** **Arnt and Miz-1 interact. A)** Schematic representation of motifs within native and mutant constructs of Arnt. The human Arnt used in this study consists of 774 amino acids and the location of its helix-loop-helix (bHLH), Per-Arnt-Sim (PAS) and the glutamine rich (Q-rich) domains are shown. The amino acid mutations in “2xmut” and “4xmut” are indicated in bold in the Helix II sequence. **B)** Miz-1/GFP and wt or mutated variants of Arnt/Flag were overexpressed as indicated. Immunoprecipitation (IP) was performed using anti-GFP and immunoblotting (IB) was performed with anti-Flag (upper panel). Input (4%) was run on a parallel gel and IB was performed with anti-Flag (middle panel). In order to verify Miz-1/GFP IP in the different samples, the co-IP membrane was stripped and incubated with anti-GFP (lower panel). **C)** HEK293 cells were co-transfected with Miz-1/Flag and Arnt/CFP. Cells were subjected to confocal microscopy to visualize Texas-red fluorescence (for Miz-1/Flag; left panel) or cyan fluorescence (for Arnt/CFP; middle panel). The right panel shows the merged image. The borders of the cytoplasm of the cells are marked in white, while the borders of nuclei are marked in yellow.

### Arnt induces reporter gene expression from the CDKN2B promoter

The *CDKN2B* promoter is an established target for the Miz-1/Myc complex. Whereas Miz-1 activates this promoter, Myc acts as a repressor through interaction with Miz-1 and displacement of p300/CBP [9,10]. To explore the possibility that Arnt might affect this Myc/Miz-1-dependent transcriptional regulation, Arnt was overexpressed in human osteosarcoma U2OS cells together with a luciferase reporter construct containing 35 nucleotides upstream of the transcriptional start site of *CDKN2B* (−35CDKN2B/luc, [25]). This construct does not contain a consensus Arnt binding site, or a canonical HRE [26]. U2OS cells are frequently used in functional studies that aim to understand the molecular mechanisms underlying hypoxic transcriptional responses as this cell line respond well to low O_2_ levels. As expected, based on the literature [14], Miz-1 induced luciferase activity from the CDKN2B promoter (Figure 2A). Likewise, Arnt caused an induction of luciferase activity from this promoter construct (Figure 2A). The stimulatory effects of Arnt and Miz-1 on this promoter construct did vary between experiments; however, we always observed significantly enhanced reporter gene activity after Arnt and Miz-1 overexpression. Mutation of the amino acids in Arnt required for Miz-1 interaction (2xmut, 4xmut) led to decreased reporter gene activity, but apparently, the low level of complex formation between Miz-1 and 2xmut Arnt and, although not detectable above the background in the co-IP assay, 4xmut Arnt was sufficient to drive reporter gene expression to a certain level in this system (Figure 2B). As stated above, Myc inhibits Miz-1 induced transcription from the *CDKN2B* promoter. The results presented in Figure 2C show that Myc also repressed Arnt-dependent reporter gene expression from this promoter, and moreover, that a mutated version of Myc that is unable to interact with Miz-1 (MycV394D) [14] failed to inhibit Arnt-induced transcription (Figure 2C). Taken together, these experiments support the concept that Arnt induces transcription from the *CDKN2B* promoter via interaction with Miz-1, and that Myc counteracts this activity through competition for the interaction surface of Miz-1.

**Figure 2:** **Arnt activates transcription from the CDKN2B promoter. A-C)** U2OS cells were transfected in 12-well plates with the reporter gene construct -35CDKN2B/Luc (300 ng) and expression plasmids encoding Miz-1 (Miz1/pcDNA) or wt Arnt (Arnt/Flag/pCMV) at the indicated concentrations **(A)**, wt Arnt or mutated variants of Arnt/Flag (Arnt (T115D/S126A)/Flag/pCMV denoted “2xmut” and Arnt (L114A/T115D/R118G/S126A) /Flag/pCMV denoted “4xmut” (100 ng each) **(B)**, and wt Arnt and wt (Myc/pcDNA3) or a mutated variant of Myc (V394D) (Myc (V394D)/pcDNA3) (100 ng each) as indicated **(C)**. The luciferase activity is presented as average +/− stdev, n = 9 in **A**; n = 6 in **B**; n = 12 in **C**. Statistical analyses: **(A)***Student’s T-test*, **(B)***ANOVA* (Bonferroni), **(C)***ANOVA* (Dunnett’s T3); ***p ≤ 0.001, ns: non significant.

### Arnt interacts with the CDKN2B promoter

To establish whether Arnt interacts with the *CDKN2B* promoter, chromatin-immunoprecipitation (ChIP) analyses combined with qPCR were performed. These experiments demonstrated that Arnt is enriched on the proximal *CDKN2B* promoter (Figure 3A) compared to a distal region of the promoter (Figure 3B) in U2OS cells. Since Arnt is an obligate partner of Hif1α and Hif2α, and thus plays an important role in hypoxia regulated gene expression [27,28], we cultured U2OS cells in 1% O_2_ for 4 or 24 hours to examine whether hypoxic conditions would affect binding of Arnt. Interestingly, recruitment of Arnt to the proximal *CDKN2B* promoter was reduced when the cells were cultured under hypoxia compared to normoxic conditions (Figure 3A). Unfortunately, with commercially available antibodies, we were not able to determine the occupation of Miz-1 on the *CDKN2B* promoter during hypoxia (or normoxia). Binding of Miz-1 to the *CDKN2B* promoter in normoxic cells has been shown previously [10,15]. As a control for hypoxia induced transcription, primers spanning the HRE in the promoter of phosphoglycerate kinase 1 (*PGK-1*) were employed to determine Arnt interaction. As reported [29], Arnt was found to bind to the HRE of *PGK-1* at normoxia, and at increased levels under hypoxic conditions (Figure 3C).

**Figure 3:** **Arnt interacts with the CDKN2B promoter.** ChIP experiments were performed on extracts from U2OS cells using an antibody (Ab) against Arnt or preimmune IgG as indicated. The cells were cultured at normoxia (21% O_2_) or at hypoxia (1% O_2_) for 4 or 24 hours before harvested. qPCR was performed with primers spanning the *CDKN2B* proximal promoter (−168/-19) **(A)**, primers spanning a distal *CDKN2B* promoter sequence (−3874/-3744) **(B)** and primers spanning a hypoxia response element (HRE) of the *PGK-1* proximal promoter (−75/+101) **(C)**. The results are given as average enrichment of the indicated promoter fragment +/− stdev, n = 6. Statistical analyses: **(A)***ANOVA* (Dunnett’s T3), **(B-C)***ANOVA* (Bonferroni); **P ≤ 0.01, *P ≤ 0.05, ns: not significant.

### Hypoxia decreases CDKN2B expression

To further explore the potential role of O_2_ pressure in the expression of *CDKN2B*, we examined whether hypoxia affected CDKN2B endogenous protein and mRNA levels. The protein level of CDKN2B decreased after 4 and 24 hours at 1% O_2_ compared to the expression at normoxia (Figure 4A). Already after 2 hours, the CDKN2B mRNA level was significantly reduced, and declined further when the hypoxic exposure was prolonged to 16 or 24 hours (Figure 4B). Thus, these results are in agreement with the ChIP results in Figure 3, and indicate that as O_2_ levels fall, Arnt is released from the promoter leading to decreased expression of *CDKN2B*. The mRNA expression of the hypoxia regulated gene PGK-1 was, in accordance with the literature [29], increased during hypoxic treatment (Figure 4C).

**Figure 4:** **Expression of CDKN2B is decreased in response to hypoxia. A-B)** U2OS cells were cultured at normoxia (21% O_2_) or at hypoxia (1% O_2_) for the time points indicated, and immunoblotting for CDKN2B **(A)** as well as qRT-PCR analyses for CDKN2B **(B)** and PGK-1 **(C)** were performed. Immunoblotting for the housekeeping protein beta-actin was used as a loading control **(A)**. The qRT-PCR values were normalized to the expression of the housekeeping gene HPRT-1, and are shown as average of relative fold change +/− stdev, three independent experiments performed in duplicates **(B and C)**. Statistical analyses: **(B)***ANOVA* (Bonferroni); **(C)***ANOVA* (Dunnett’s T3); ***p ≤ 0.001, *P ≤ 0.05, ns: non significant.

### Repression of Arnt, Miz-1 and Hifα causes downregulation of CDKN2B mRNA levels

Expression of siRNA against Arnt (siArnt) caused a significant decrease in the CDKN2B mRNA expression, further supporting a role for Arnt in transcriptional regulation of this gene (Figure 5A, compare columns 1 and 3). As expected from previous studies [9,10], inhibition of Miz-1 also repressed the expression of *CDKN2B* (Figure 5A, compare columns 1 and 5). Intriguingly, knockdown of Hif1α and Hif2α also caused reduced CDKN2B mRNA levels at normoxia (Figure 5A, compare column 1 with column 7 and 9). The effect of siHif1α was significant, despite the fact that the level of Hif1α protein at normoxia was below the detectable threshold (Figure 5C, right upper panel). In contrast, Hif2α was readily detectable at normoxia in this cell line (Figure 5C, right lower panel), as has also been reported previously [30]. In agreement with the results in Figure 4, hypoxic treatment for 6 hours decreased CDKN2B mRNA levels with around 50-60% in presence of control siRNA (Figure 5A, compare columns 1 and 2), and administration of siRNA against Arnt, Miz-1 and Hif2α under hypoxic conditions further repressed *CDKN2B* expression (Figure 5A, compare lane 2 with lanes 4, 6 and 10). In contrast, siHif1α had no significant effect under hypoxic conditions compared to control siRNA (Figure 5A, compare lanes 2 and 8).

**Figure 5:** **Inhibition of Miz-1, Arnt and Hifα expression reduces CDKN2B mRNA levels. A-C)** U2OS cells were transfected with siRNA (10 nM) against Arnt, Miz-1, Hif1α and Hif2α as indicated and cultured at normoxia (21% O_2_) or hypoxia (1% O_2_) for 6 hours. **A)** qRT-PCR analyses of CDKN2B mRNA levels after administration of the different siRNAs are presented as relative fold changes compared to control siRNA at normoxia (column 1). **B)** qRT-PCR analysis of mRNA expression of Arnt, Miz-1, Hif1α and Hif2α after siRNA treatment. The mRNA levels after administration of the different siRNAs are presented as relative fold changes compared to control siRNA at normoxia for each specific mRNA species. **C)** Protein levels of Arnt (upper left panel), Miz-1 (lower left panel), Hif1α (upper right panel) and Hif2α (lower right panel) in response to siRNA treatment and hypoxia were determined by immunoblotting. Immunoblotting for beta-actin was included to control for protein loading. **D)** U2OS cells were cultured at normoxia (21% O_2_) or at hypoxia (1% O_2_) for the time points indicated, and qRT-PCR analyses for Miz-1 mRNA expression were performed. The qRT-PCR values in **A**, **B** and **D** were normalized to the housekeeping gene HPRT-1, and are shown as average of two or three independent experiments performed in duplicates (n = 4 for **A** and **B**, n= 6 for **D**). **E)** U2OS cells were transfected with siRNA (10 nM) against Miz-1, Hif1α and Hif2α or a negative control siRNA together with the −35CDKN2B/luc reporter (300 ng) in the presence or absence of an Arnt expression vector (Arnt/Flag/pCMV, 100 ng) as indicated. The luciferase activity is presented as average +/− stdev, n = 3. Statistical analyses: **(A-B and E)***Student’s T-test*, **(D)***ANOVA* (Bonferroni); ***p ≤ 0.001, **P ≤ 0.01, *P ≤ 0.05, ns: non significant.

Intriguingly, we found that Miz-1 mRNA levels were suppressed in response to hypoxia (Figure 5B compare lanes 5 and 6), as was the protein level (Figure 5C, left lower panel). A comparable response was observed when endogenous Miz-1 mRNA expression was determined in response to hypoxia (Figure 5D), suggesting that this gene is regulated by O_2_ tension and substantiating the impact of Miz-1 as an important activator of *CDKN2B* in the normoxic state. This effect might be cell line specific, however, as a similar downregulation of Miz-1 mRNA in response to hypoxia is not observed in HCT116 or WT-8 cells [22]. The gene encoding Miz-1 contains an HRE element in the 5’ untranslated region as well as in intron 1, and it remains to be determined whether HIFs interact with these sequences. The mRNA levels of Arnt and Hif1α were also slightly reduced in response to hypoxia (Figure 5B, compare lanes 1 and 2 for Arnt and lanes 9 and 10 for Hif1α). However the corresponding protein levels increased, as they did for Hif2α, and as previously reported [31]. These results suggest that the Arnt/Miz-1 complex, possibly in association with Hifα, is involved in *CDKN2B* gene regulation in U2OS cells. Further supporting the scenario that such a complex has impact on transcription from the *CDKN2B* promoter are the results shown in Figure 5E, namely that Arnt-induced *CDKN2B-*promoter dependent luciferase expression is inhibited as a consequence of repressing Miz-1, Hif1α or Hif2α. All factors were relatively efficiently repressed by the corresponding siRNA, both at the mRNA level and at the protein level (Figure 5B and C).

### Hypoxia leads to release of Myc from the *CDKN2B* promoter

Since Myc is an established inhibitor of *CDKN2B* expression, we hypothesized that Myc might replace Arnt on the proximal promoter during hypoxia. In contrast to our theory, however, ChIP experiments demonstrated decreased enrichment of Myc in response to low O_2_ pressure (Figure 6A, left panel). Actually, it was previously reported that Myc is released from the *CDKN2B* promoter in hypoxic cells, as well as from the *CDKN2A* promoter, which was used as a control in our experiment (Figure 6B and [22]). *CDKN2B* is under tight transcriptional control by multiple signaling cascades, transcription factors and epigenetic mechanisms [32,33], and most likely, other transcription pathways than those investigated in the present study are involved in the repression of this gene at hypoxic conditions.

**Figure 6:** **Hypoxia leads to release of Myc from the *CDKN2B *promoter.** ChIP experiments were performed on extracts from U2OS cells using an antibody (Ab) against Myc or preimmune IgG as indicated. The cells were cultured at normoxia (21% O_2_) or at hypoxia (1% O_2_) for 4 or 24 hours before harvested. qPCR was performed with primers spanning the proximal (−168/-19) (**A**, left panel) or distal (−3874/-3744) (**A**, right panel) *CDKN2B* promoter sequences, and primers spanning either the proximal (+6/+106) (**B**, left panel)) or distal (−2337 /-2158) (**B**, right panel) *CDKN1A* promoter sequences. The results are given as average enrichment of the indicated promoter fragment +/− stdev, n = 6. Statistical analyses: *ANOVA* (Dunnett’s T3), **P ≤ 0.01, *P ≤ 0.05, ns: not significant. For the IgG control experiments there were no statistically significant differences detected, apart from on the *CDKN2B* distal promoter, as indicated in the figure (**A**, right panel).

## Discussion

Transcriptional signaling induced by low O_2_ tension and irregular Myc expression play crucial roles in tumor development and cancer progression [18,20]. Both pathways affect cell proliferation and survival, and the associated transcriptional regulators converge on promoters of several genes encoding cell cycle regulatory factors [22,34-38]. It has been suggested that Hif1α counteracts Myc on the proximal promoters of *CDKN1A*, *CDKN1B* and *CDKN2B* by disrupting the complex formation between Myc/Max and Miz-1 [22,38]. In contrast, Hif2α enhances Myc activity from these promoters in a renal clear cell carcinoma cell line overexpressing the von Hippel Lindau factor (WT-8 cells, [22]). The DNA binding domain of Hifα appears not to be required for these actions, but the underlying biochemistry is not well understood.

The data presented in this study demonstrate that Miz-1 and Arnt can reside in the same protein complex. Moreover, we show that Arnt is enriched on a promoter that is well documented as a Myc/Miz-1 target [10] and that this promoter is regulated by hypoxia. These findings are important as they define a direct physical protein interaction that integrates these two pathways that are recurrently dysregulated in cancer cells. Interestingly, our mutational analyses suggest that Arnt provides a similar interaction surface for Miz-1 as Myc does [14]. Miz-1 interacts with different types of proteins [15,16,39], but to our knowledge, Arnt is the only bHLH factor demonstrated to interact with Miz-1 besides Myc. Although we were unable to map the domain of Miz-1 required for interaction with Arnt, we anticipate a similar mode of interaction as for the Myc/Miz-1 complex, with the further implication that Myc and Arnt might compete for Miz-1 interaction. This assumption is supported by the observation that Arnt-induced transcription from the *CDKN2B* promoter was suppressed by wild type Myc, but not by a mutated form (V394D) that is unable to interact with Miz-1, as shown previously [13,14]. A potential mutual exclusive interaction of Arnt and Myc with Miz-1 on common target genes might have considerable functional cellular consequences.

Myc is in complex with Max when it interacts with Miz-1, and comparably our results possibly suggest that activation by Arnt on the *CDKN2B* promoter is dependent on Hifα, as knockdown of Hifα caused decreased transcriptional capacity by Arnt. The amino acid composition of helix II in Hif1α and 2α does not suggest that they can interact directly with Miz-1 in a similar fashion as Arnt and Myc. We regard it as plausible therefore that regulation of CDKI encoding genes by Hifα generally is dependent on a complex formation between Arnt and Miz-1 (although we were unable to detect a complex consisting of all three factors in co-IP experiments). Interestingly, Arnt has been implicated in the transcriptional regulation of several CDKIs [36,40], of which the majority is also regulated by Miz-1 [15,41]. For instance, Arnt induces expression of *CDKN1B*, an established Myc/Miz-1 target gene [15], under hypoxic conditions [36]. Likewise, in hepatocellular carcinoma cells (HCC), Arnt up-regulates *CDKN1C*[40], a gene that is also regulated by the Myc/Miz-1 complex [41]. Together with the present study, these studies suggest that Arnt, via complex formation with Miz-1, may function as a general anchor for Hifα on CDKI promoters.

Based on our results we propose the following hypothesis (Figure 7): In U2OS cells, and perhaps in other cancer cells with dysregulated proliferation, we envision that under normoxia, a transactivating complex consisting of Miz-1/Arnt and perhaps Hif1α or Hif2α is anchored on the *CDKN2B* proximal promoter via the DNA binding domain of Miz-1, stimulating expression of CDKN2B. Hypoxia response elements are not required for Arnt/Hifα complex binding to occur. A transrepressive complex consisting of Miz-1 and Myc/Max will counteract the activation mediated by the Miz-1/Arnt complex, and we suggest that the opposite actions of these complexes ensure adequate levels of CDKN2B in normoxic cells. Upon hypoxia, the majority of the transactivating Arnt/Hifα complexes are released from the *CDKN2B* promoter, leading to decreased expression. Similarly, Myc is released from the promoter, and might therefore not be essential for transcriptional repression from this promoter in the hypoxic state, as it indeed is in normoxic cells (our results and [10]). Of note is that Gordan et al. reported that in hypoxic colorectal cancer cells (HCT116), Myc is released from several CDKI promoters, among them CDKN2B [22]. The reduced expression of Miz-1 at low O_2_ pressure should also contribute to lower CDKN2B expression, both because of its role as a transactivator and because the recruitment of Arnt will be diminished. Future experiments will establish if Miz-1 is present at the *CDKN2B* promoter at hypoxia, influenced by yet unidentified repressive factors, or whether Miz-1 independent mechanisms are responsible for decreased CDNK2B expression as O_2_ levels falls. The potential biomedical modifications that cause the release of the Arnt/Hifα and Myc/Max complexes from the *CDKN2B* promoter during low oxygen conditions remain to be determined. The release might be regulated by diverse posttranslational modifications, e.g. oxygen-dependent hydroxylation, histone-modifying mechanisms like de-acetylation and/or by cofactor interactions, as have been described for other promoters regulated by Myc or Hifα [6,42,43].

**Figure 7:** **Model based on the presented data.** We hypothesize that in U2OS cells under normoxia, a complex consisting of Miz-1/Arnt and Hif1α and/or Hif2α is anchored to the *CDKN2B* proximal promoter via Miz-1. A repressive complex of Myc/Max, which competes for the same interaction surface on Miz-1, counteracts this activity, and the mutually exclusive interaction of these complexes ensures adequate levels of CDKN2B at normoxia (left). Upon hypoxia, the examined complexes binding at high O_2_ pressure leave the *CDKN2B* promoter, allowing yet unknown factors to interact with Miz-1 or to act by other means to repress the expression of CDKN2B (right).

Our findings that Arnt activates the CDKN2B promoter and that knockdown of Arnt causes a decrease in the mRNA level of CDKN2B in U2OS cells are in line with recent findings in HCC [40]. This study suggested that Arnt-dependent regulation of cell cycle proteins, among them CDKN2B, causes HCC stagnancy and decreased metastasis and that high intratumoral Arnt expression is correlated with increased overall survival and reduced recurrence incidence of HCC patients [40]. CDKN2B also acts as a tumor suppressor in other cancer types [44,45]. However the role of Arnt in regulation of CDKN2B in these cancer types remains to be examined. Up-regulation of CDKIs in response to hypoxia restricts cell proliferation in a variety of cancer cell lines, including U2OS cells [31,35,36,46-48], and Arnt has been implicated in induced expression of CDKN1B under hypoxic conditions [36]. Our finding that Arnt is released from the *CDKN2B* promoter in response to hypoxia, followed by reduced CDKN2B expression is therefore somewhat contradictory to the overall effects of hypoxia on proliferation in U2OS cells. However, CDKN2B is also repressed at low O_2_ levels in HCT116 cells [1], although hypoxia induces cell cycle arrest in these cells [38], suggesting that it is the combined transcriptional changes in cell cycle regulatory factors that will determine the final proliferative characteristics of a tumor cell. Intriguingly, the relative expression of Hif1α and 2α might also affect the proliferation rate [22]. Taken together, the wealth of studies that exist on CDK-inhibitors in cancer cell lines clearly point to that expression of these proteins is differently regulated in different cell lines [31,35,36,46-48]. Although this study was limited to U2OS cells, we envision that the interaction between Miz-1 and Arnt might be of importance in cell cycle progression in other cancer cells, however not necessarily for the regulation of CDKN2B. These cell-type and gene-specific effects are intriguing and possibly reflect the many different ways cancer cells adapt in order to survive, and underscore the necessity to analyze the molecular pathways controlling cell cycle progression in diverse biological settings.

## Conclusions

In conclusion, our finding that Arnt and Miz-1 reside in the same protein complex directly integrates hypoxia and Myc-dependent signaling pathways. This direct link between the HIF and Myc pathways may have important implications for understanding their roles in cell cycle progression and cancer development.

## Methods

### Plasmid constructs

The mutations in helix II of Arnt, T115D/S126A denoted “2xmut” and L114A/T115D/R118G/S126A denoted “4xmut”, were constructed using the Quick Change XL Site-directed Mutagenesis Kit (Stratagene). ArntΔbHLH (deleted of amino acids 67–146) has been described previously [49,50] as has the plasmid Arnt/pECFP-C1 [51] and the luciferase reporter construct -35CDKN2B /Luc [25] (kindly provided by Dr. XF Wang (Pharmacology and Cancer Biology, Duke University School of Medicine, Durham, NC, USA). Myc/pcDNA3 was kindly provided by Dr. F. Haenel (Hans-Knöll-Institut für Naturstoff-Forschung, Department of Cell and Molecular Biology, 07745 Jena, Germany), and Miz-1/pcDNA3 by Dr. L.G. Larsson (Department of Microbiology, Tumor and Cell Biology, Karolinska Institutet, Stockholm, Sweden).

### Yeast two-hybrid assay

The Matchmaker GAL4 Two-hybrid System 3 (Clontech) was used to identify Arnt-interacting proteins from a cDNA library prepared from Y1 mouse adrenocortical tumor cells using the pCMV-ScriptXR cDNA library construction kit (Agilent Technologies, Stratagene Products Division). Arnt deleted of its transactivation domain (Q) was fused to the GAL4 DNA-binding domain of pGBKT7 (ArntΔQ/pGBKT7, amino acid 1–618). The Y1 cDNA-library was expressed as fusion proteins with the GAL4 activation domain of pGADT7. The *Saccharomyces cerevisiae* strain AH109 was transformed with the plasmids and positive clones were selected based on their ability to grow at high stringency on synthetic dropout plates lacking adenine, leucine, tryptophan and histidine. To verify for protein interactions the positive colonies were restreaked on selection media as described in the manufactures protocol (Matchmaker GAL4 Two-hybrid System 3, Clontech).

### Cell cultures

The human osteosarcoma U2OS (ATCC: HTB-96™) and HEK293 (ATCC: CRL-1573™) cell lines were cultured in high glucose DMEM (D5786, Sigma) supplemented with 10% bovine calf serum, penicillin (100 units/ml) and streptomycin (100 mg/ml) (Sigma). The HEK293-EBNA cell medium was supplemented with 25 mM HEPES. The cells were maintained in 5% CO_2_ humidified atmosphere at 37°C. For hypoxic condition, the cells were cultured at 1% O_2_ for the time points indicated in the figures.

### Cell transfection

For transient transfection experiments, U2OS cells were plated at a density of 6.5×10^4^ cells per well onto 12-well plates and transiently transfected the following day using XtremeGene9 (Roche). Cells were transfected with reporter plasmid (0.3 μg, −35CDKN2B/Luc) and expression plasmids (0.1 ug) as indicated in the figures. The total amount of DNA was kept constant by compensating with the plasmid psp70 (New England Biolabs). 24 hrs after transfection start, the cells were washed once with PBS and lysed in luciferase lysis buffer (10 mM Tris–HCl pH 8.0, 4 mM EDTA, 150 mM NaCl, 0.65% NP40). Cell extracts were then assayed for luciferase activity on a LUCY-3 luminometer (Anthos, Austria). Co-immunoprecipitation (co-IP) assays were conducted using Cos-1 cells. The cells were grown in 100 mm dishes to 70–80% confluency and transfected with indicated plasmid combinations using X-tremeGene 9 (Roche). The manufacture’s protocol was followed using a total amount of 5 μg plasmid per dish. Transfected cells were incubated for 36 hours at 5% CO_2_ in 37°C before preparation of whole cell extract. The cells were washed with ice-cold PBS before lysis buffer (25 mM Hepes, 100 mM NaCl, 5 mM EDTA, 20 mM glycerol phosphate, 0.5% Triton, 20% glycerol; 300 μl) containing protease inhibitors (100 μM (Na_3_VO_4_), 2 mM DTT, 1 mM PMSF, 5 μg/μl aprotinin and 5 μg/μl leupeptin)) was added. The extracts were then sonicated (2 × 5 sec/amplitude 40), and centrifuged at 13000 rpm (16000 × g) for 5 minutes at 4°C to pellet cell debris. The supernatants were stored at −80°C.

### Co-immunoprecipitation assay

Cell lysates (800 μg total protein in a volume of 400 μl lysis buffer; see above) were pre-cleared with recombinant Protein G Agarose (10 μl, cat #15920-010, Invitrogen). Anti-GFP saturated rProtein G Agarose was prepared by incubating 50/50 rProtein G Agarose/TBS slurry (800 μl) with anti-GFP (56 μg) and incubated for 2 hours on a rotation platform at 4°C. The precleared extracts were then incubated with the anti-GFP saturated rProtein G-Agarose on a rotating platform o/n at 4°C. The beads were vigorously washed three times with ice-cold lysis buffer. 2× loading buffer (30 μl; 125 mM Tris–HCl pH 6.8, 4% (w/v) SDS, 20% (w/v) Glycerol and 0.004% (w/v) BromPhenol Blue) was added to the beads and the samples were incubated at 95°C for 5 minutes. Proteins were resolved by 8% SDS-PAGE and subjected to immunoblotting.

### Immunoblotting

The co-IP membranes were incubated with Flag antibody (1/3000, diluted in 1× PBS-T (0.1% (v/v) Tween in 1 × PBS), (M2; Stratagene)) or GFP antibody (1/3000, diluted in 1 × PBS-T, (JL*-*8; BD Biosciences)), and subsequently with an HRP-conjugated goat anti-mouse secondary antibody (1/10000 in 1× PBS-T) using the Supersignal Chemoluminiscent substrate (Thermo scientific) for detection. For visualization of the immunostaining patterns, the membranes were immediately exposed in a Luminescent Image analyzer (LAS 3000, Fujifilm) for 1–15 minutes. Protein levels of Arnt, Miz-1, Hif1α and Hif2α upon their downregulation by specific siRNA were also analysed by immunoblotting using antibodies against Arnt [52], Miz-1 (Santa Cruz), Hif1α (Abcam), Hif2α (Abcam) and beta-actin (Abcam). CDKN2B expression was detected using the C-20 antibody from Santa Cruz (sc-612).

### Cellular localization assay

The assay was performed essentially as described [51]. Briefly, HEK293 cells were grown on cover slips and transfected with the expression plasmids Flag/Miz-1 and pECFP/Arnt using the Lipofectamine Reagent (Invitrogen). 24 hours after transfection, cells were fixed in 4% paraformaldehyde/PBS for 15 min at RT. Blocking was performed with 10% FBS/PBS for 15 min at RT. Cells were then subjected to incubation with anti-Flag [1:100 (M2; Stratagene) in 1% BSA/0.1% Triton-X100/PBS] and Texas-red conjugated goat anti-mouse antibody (Molecular Probes). Cells were washed 4× for 10 min with PBS and subjected to confocal laser scanning microscopy.

### Chromatin immunoprecipitation assay (ChIP)

U2OS cells were cultured at 21% O_2_ or reduced O_2_ (1% O_2_) for 4 or 24 hours, and ChIP analyses combined with quantitative PCR were performed as previously described [53] using antibodies against Arnt [52], Myc (Santa Cruz) or IgG (Jackson ImmunoResearch). PCR primers flanking the proximal promoter of the *CDKN2B* gene (−168/-19) were F: 5′- cgcatgcgtcctagcatctttg -3′ and R: 5′- gaattccgttttcagctgggcc -3′ giving a product of 149 bp. Distal *CDKN2B* promoter primers (−3874/-3744) were F: 5′- ggtgggccctaatccaatctgac -3′ and R: 5′- gcacatggccatcctactgctg -3′ giving a product of 130 bp (see [25] for nucleotide numbering of the *CDKN2B* promoter). PCR primers flanking the proximal promoter of the *CDKN1A* gene (+6/+106) were F: 5′- tgtgtgagcagctgccgaagtc -3′ and R: 5′- tgccgccgctctctcacct -3′ giving a product of 100 bp. Distal *CDKN1A* promoter primers (−2337 /-2158) were F: 5′- catccctatgctgcctgcttcc -3′ and R: 5′- cctgtctcctaccatccccttcct -3′ giving a product of 179 bp. Primers spanning the HRE site of the *PGK-1* promoter (−75/+101) were F: 5′- gacagcgccagggagcaatg -3′ and R: 5′- gct ccggaggcttgcagaatg -3′ giving a product of 176 bp. The comparative Ct method was used for relative quantification of target DNA amplification using SYBR Green.

### RNA interference experiment

U2OS cells were transfected with control siRNA (10 nM; 5′- UUCUCCGAACGUGUCACGU -3′) or siRNA against Arnt (5′-GGAACAAGAUGACAGCCUATT -3′), Miz-1 (5′- GCCUCAUCAGCCUGCUGAATT -3′), Hif1α (5′- GAAGAACUAUGAACAUAAATT -3′) and Hif2α (5′- CGGAUAGACUUAUUGCCAATT -3′) (Qiagen) using the HiPerFect transfection reagent (Qiagen) according to the manufacturer’s instructions. The cells were cultured for 48 hours and then placed at 21% or 1% O_2_ for 6 hours before harvested.

### Quantative RT-PCR

RNA was prepared from U2OS cells using Trizol (Life Technologies). RNA (1 μg) was reversely transcribed using Superscript II Reverse Transcriptase kit (Life Technologies) according to the manufacturer’s recommendations. TaqMan quantitative RT-PCR was performed using the ABI 7300 system with TaqMan master mix and pre-design primer/probes for human Arnt, Miz-1, Hif1α and Hif2α (Arnt: cat# Hs01121918_m1, Miz (ZBTB17) cat#: Hs01114794_g1, HIF1α cat#: Hs00153153_m1, HIF2α cat#: Hs01026142_m1, CDKN2B cat#: Hs00793225_m1, PGK-1 cat# Hs00943178-g1, HPRT cat#: 4326321E; Applied Biosystems). Hypoxanthinephophoribosyltransferase (HPRT) was used as an endogenous control in ∆∆CT analyses. All measurements were performed twice in duplicates.

### Statistics

One-way analysis of variance (ANOVA) followed by Bonferroni adjustment was used for multiple comparisons of data presented in Figures 2B, 3B, 4B and 5D. ANOVA with Dunnett’s T3 adjustment was used when variances were unequal (Figures 2C, 3A and C, 4C, 6A and B). *Student’s t-test* was used in Figures 2A, 5A, B and E.

## Abbreviations

Arnt: Aryl hydrocarbon receptor nuclear translocator; ChIP: Chromatin immunoprecipitation assays; co-IP: Co-immunoprecipitation; CDK: Cyclin-dependent kinase; CDKI: Cyclin-dependent kinase inhibitor; CDKN2B: Cyclin-dependent kinase inhibitor 2B; DMEM: Dulbecco’s modified Eagle’s medium; EDTA: Ethylenediaminetetraacetic acid; GFP: Green fluorescent protein; HCC: Hepatocellular carcinoma cells; HEPES: 4-(2-hydroxyethyl)-1-piperazineethanesulfonic acid; HIF: Hypoxia-inducible factor; HLH: Helix-loop-helix; HRE: Hypoxia response element; HPRT: Hypoxanthinephophoribosyltransferase; INR: initiator; Miz-1: Myc-interacting zinc finger protein 1; PAS: Per-Arnt-Sim factors; PBS: Phosphate buffered saline; PGK-1: Phosphoglycerate kinase 1; PMSF: Phenylmethanesulfonylfluoride; SDS: Sodium dodecyl sulfate.

## Competing interests

The authors have no competing interests to declare.

## Authors’ contributions

RA, KG, KSA, JLR, LP and MB conceived and designed the experiments. RA, KG, KSA, EAH and JLR performed the experiments. All authors analyzed and interpreted data. RA, KG and MB drafted the manuscript. All authors critically revised the manuscript. All authors have approved the final manuscript.
